The article "Accessing the Inaccessible: Redefining Play as a Spectrum" was published in 2018. Journal: Front Psychol.

# Accessing the Inaccessible: Redefining Play as a Spectrum

**DOI:** 10.3389/fpsyg.2018.01124

**Published:** 2018-08-02

**Authors:** Jennifer M. Zosh, Kathy Hirsh-Pasek, Emily J. Hopkins, Hanne Jensen, Claire Liu, Dave Neale, S. Lynneth Solis, David Whitebread

**Affiliations:** ^1^The Pennsylvania State University Brandywine, Media, PA, United States; ^2^Department of Psychology, Temple University, Philadelphia, PA, United States; ^3^The Brookings Institution, Washington, DC, United States; ^4^The LEGO Foundation, Billund, Denmark; ^5^Graduate School of Education, Harvard University, Cambridge, MA, United States; ^6^School of Education, University of Delaware, Newark, DE, United States; ^7^Homerton College, University of Cambridge, Cambridge, United Kingdom

**Keywords:** play, playful learning, cognitive development, children, games, pedagogy

## Abstract

Defining play has plagued researchers and philosophers for years. From describing play as an inaccessible concept due to its complexity, to providing checklists of features, the field has struggled with how to conceptualize and operationalize “play.” This theoretical piece reviews the literature about both play and learning and suggests that by viewing play as a spectrum – that ranges from free play (no guidance or support) to guided play and games (including purposeful adult support while maintaining playful elements), we better capture the true essence of play and explain its relationship to learning. Insights from the Science of Learning allow us to better understand why play supports learning across social and academic domains. By changing the lens through which we conceptualize play, we account for previous findings in a cohesive way while also proposing new avenues of exploration for the field to study the role of learning through play across age and context.

The most irritating feature of play is not the perceptual incoherence, as such, but rather, that play taunts us with its inaccessibility. We feel that something is behind it all, but we do not know, or have forgotten how to see it. [scholar Robert Fagen (1981) as cited in Sutton-Smith, 1997].

Play is a roomy subject, broad in human experience, rich and various over time and place, and accommodating pursuits as diverse as peekaboo and party banter, sandlot baseball and contract bridge, scuba diving and Scrabble. Play welcomes opposites, too. Play can be free—ungoverned by anything more complicated than choosing which stick is best to improvise a light saber—or fixed and codified, as in those instances when soccer players submit to scrupulous “laws.” Play can take active or passive form and can be vicarious or engaging—and so we recognize play in both the spectator and the actor (Eberle, 2014, p. 214).

Play is often defined as activity done for its own sake, characterized by means rather than ends (the process is more important than any end point or goal), flexibility (objects are put in new combinations or roles are acted out in new ways), and positive affect (children often smile, laugh, and say they enjoy it). These criteria contrast play with exploration (focused investigation as a child gets more familiar with a new toy or environment, that may then lead into play), work (which has a definite goal), and games (more organized activities in which there is some goal, typically winning the game) (Smith and Pellegrini, 2013).

For something so easy to observe, that occurs in monkeys, humans and even octopuses (Burghardt, 2011), play has been notoriously difficult to define. An infant playing with vocalizations while engaged in primary interactions with his parent is engaged in play, as is a 7-year-old deeply focused on a game of checkers. Children can play by themselves or with a group of 15 others.

The widely variable, inaccessible nature of play has not been lost on those writing on the topic. As the quotes above exemplify, play is complex. And a number of researchers have attempted an all-encompassing operational definition of the construct. For instance, Vygotsky (1967) stressed that, through sociodramatic play in particular, both children’s cognitive development and higher mental functions (e.g., inhibition) are strengthened as they navigate through the play situation and operate within the zone of proximal development (see Bodrova and Leong, 2015 for a review). Piaget (1962), however, focused on play for its own sake and conceptualized play as the way that children assimilated the external world to match their own concepts rather than to learn something new. Stuart Brown (2010) argues that play is evolutionary and has the following properties: apparently purposeless/done for its own sake, voluntary, inherent attraction, freedom from time, diminished consciousness of self, improvisational potential, and continuation desire. Gray (2013) also provides a list of features to describe play, with some overlap. His conceptualization maintains that play (1) is directed and chosen by the child, (2) is as an activity in which the focus is not the end-state or a goal, but the means themselves, (3) consists of structure that comes from the minds of the players and not external constraints, (4) is imaginative and separate from real life and, (5) involves mental, non-stressed activity.

Garvey (1990) joins in with a list of characteristics that has been widely cited suggesting that play is pleasurable, with no extrinsic goals, spontaneous and voluntary, involves engagement on the part of the player, and also that it is related to other cognitive and social functions that exist outside of play. Similarly, Smith and Pellegrini (2013) suggest that play is activity that is done with no extrinsic goal with the focus being the play itself, is flexible, and involves positive affect. They separate play from exploration and games. Weisberg et al. (2013) used previous research (Garvey, 1990; Sutton-Smith, 1997; Johnson et al., 1999; Hirsh-Pasek and Golinkoff, 2003; Hirsh-Pasek et al., 2009; Pellegrini, 2009; Burghardt, 2011; Fisher et al., 2011) to suggest four criteria that emerge in the flood of definitions to demarcate whether or not an activity is play. Play (1) has to have no specific purpose nor be linked to survival, (2) can oftentimes be exaggerated – e.g., playful experiences often are not necessarily related to how things work in regular, everyday life, (3) requires both joyful and voluntary participation, and (4) is child-led, not adult-directed.

Though it is easy to find the overlap, these should not mask key points of disagreement, especially when it comes to the purpose of play and the role of structure or scaffolding from others. For example, the idea that play requires that there is no goal, suggests that children playing a pretend play scenario that was crafted to build vocabulary is not play, even if the children are leading their exploration and having fun pretending to be at a grocery store. It suggests that children playing a board game are not really playing. Further, child-directed play would lose its cache as play if adults suggested that the children become explorers who hunted down magic bugs in the backyard. These conceptual differences lead to definitional confusion within the fields of education and developmental psychology. The criterial features of play are hard to pin down.

In this piece, we suggest a reason why discussions of play are often vague and conclude that broad definitions of the construct are too encompassing and as such, void of the nuance that this field demands. Rather than holding to one set of criteria, it might be better to conceptualize play as unfolding along a spectrum, or continuum, that ranges from free play, captured in definitions provided by Garvey (1990), Pellegrini (2009), Stuart Brown (2010), and Weisberg et al. (2013), to forms of play that are none-the-less child directed but that have inherent goals like guided play, and games (Hassinger-Das et al., 2017). Defining play as a continuum might also allow us to better specify not only the types of play, but the outcomes that emerge from each genre. For example, free play, with no extrinsic goal, might prove optimal for social development whereas guided play, in which adults take supportive (rather than leading) roles in service of a learning goal is repeatedly demonstrated to be effective for more academic types of learning. Here we attempt to chart a definition of play that allows us to capture the Play Spectrum and thus to make more refined hypotheses about how play relates to varied aspects of development – from traditional academic outcomes to the newer conceptualizations of skills needed for 21st century success [e.g., Golinkoff and Hirsh-Pasek’s (2016) 6C’s: collaboration, communication, content, critical thinking, creative innovation, and confidence].

Thinking about play as a spectrum enables us to retain a play essence where children experience joy and have agency in their play contexts while also recognizing that play may take many different forms and serve many different functions. We acknowledge that while there is little disagreement in the function of play as an avenue for social interaction and enjoyment, there is disagreement about the functions of play for learning. Here, we first review the range of experiences that would fall along our proposed play continuum, taking a more bird’s eye view of the literature while suggesting that this more nuanced view provides cohesion amongst seemingly contradictory views of play. Then, we will use evidence generated from the Science of Learning, a multi-disciplinary approach that seeks to characterize how learning occurs and is supported through lessons learned across education, machine learning, linguistics, cognitive science, neurobiology, psychology, and other fields (Bransford et al., 1999) to spotlight guided play as a context that clearly demonstrates learning through play, but would not technically fit the global definition of play by Pellegrini and others. Finally, we end with the suggestion that a more inclusive and nuanced understanding of play allows the field to better understand findings to date about play and learning and generate new hypotheses moving forward.

## A More Nuanced Definition of Play

Free play, in which adults do not guide or scaffold, and in which there is no goal, is often hailed as the gold standard of play and is the focus of most of the traditional definitions we mentioned above (Gray, 2013). During free play, the child initiates and directs play. This happens when children sit in front of a mountain of building blocks that are not designed to build a particular outcome, or when children construct a fort in the living room. There is no pre-determined learning goal. There is a large body of research on how this type of play may benefit children and lead to positive developmental outcomes. But this laser-focus on one type of play prevented scholars and researchers from examining a wider range of experiences that are adult-scaffolded but remain playful in essence.

We argue that one can begin to add more specificity and nuance to the definition of play by imagining free play as one end of a spectrum (see **Figure 1**). In effect, we attempt to answer the call of Pyle et al. (2017) for “a need to move away from a binary stance regarding play and toward an integration of perspectives and practices, with different types of play perceived as complementary rather than incompatible” (p. 311). In free play, the child initiates the play context and also directs the play within that context. In contrast, if the adult chooses or arranges a context for learning, but the child directs the play within that context, we have guided play. Guided play can take the form of an adult playing with a child and offering scaffolding and guidance or an adult setting up a space or activity in such a way as to provide support as a child plays on their own (e.g., games). Children’s museums are an excellent example of the latter (see Sobel and Jipson, 2016 for a review). Guided play differs from free play in two ways: an adult helps to structure the activity, and the activity is centered around a learning goal. Critically, however, the child must still retain agency to direct the activity.

**FIGURE 1:** Play conceptualized as a spectrum captures playful experiences that differ along a continuum in terms of initiation and direction of the experience and whether or not there is a learning goal.

If a child initiates a context for play and then an adult intervenes to direct the play within that context, we enter co-opted play, not guided play. The child might have been interested in building a circus out of blocks, yet the well-intentioned parent swept in to declare that the animals were at the zoo, redirecting the child’s vision and robbing her of some agency in the play experience. When adults initiate and direct using playful elements, the scene more closely resembles direct instruction – even if it is dressed up in playful “clothing.” Habgood and Ainsworth (2011) cite Bruckman’s (1999) term of “chocolate covered broccoli.” Here a well-meaning adult decides that today, her child is learning about shapes and that she will be sure that she keeps the child on task by arranging the different shapes, counting sides, encouraging the child to place the blocks in appropriately shaped holes, and misses the opportunity to go on a “shape hunt” around the house.

The idea that discovery-based, active learning might prove a powerful pedagogical approach has been discussed for some time (e.g., Hirsh-Pasek et al., 2009; Bonawitz et al., 2011). Alfieri et al. (2011) conducted a meta-analysis of 164 studies and found that assisted discovery methods (those similar in nature to guided play in which adults support but children lead) resulted in the best learning outcomes (in domains as varied as: math, computer skills, science, physical/motor, and verbal and social skills) when compared to either free play or direct instruction. Research over the last few decades (see Hirsh-Pasek et al., 2015 for a review) has repeatedly shown that learning is optimized when adults scaffold an environment or feedback toward a learning goal but the learning environment encourages fun child-led exploration and discovery.

The expansion of our definition of play to include guided play widens the range of contexts and topic areas where play might have a beneficial impact on learning. Research in the past has found that free play was less effective in academic settings than direct instruction (Pianta et al., 2009; Fuller et al., 2017), but that does not mean that playful learning has no place in education. Rather, guided play, with its adult support and focus on particular learning goal, may offer an optimal pedagogical approach in academic contexts. In domains ranging from STEM [spatial thinking (Fisher et al., 2013)] to literacy (Han et al., 2010; Nicolopoulou et al., 2015; Hassinger-Das et al., 2016; Cavanaugh et al., 2017; Toub et al., 2018), children perform better in guided play than in free play and equal to or better than in direct instruction (though see Jirout and Klahr, 2012). Even studies of causal reasoning in infancy echo this idea. Work by Sim and Xu (2015) finds that 19-month-old toddlers are more likely to figure out what caused a machine to activate and to generalize that causal information in a guided, but not free play, condition.

## Lessons From the Science of Learning

### Why Guided Play Primes Learning

In 2015, several of the authors of this piece suggested that the science of learning – a newly minted amalgamation of research in psychology, education, neuroscience, machine learning, linguistics and others – has reached some consensus on features that comprise optimal learning environments (Hirsh-Pasek et al., 2015). Though first presented in the context of app use with education goals, the features that optimize learning processes are context general rather than task specific. In this piece, it was suggested that children learn best when the learning is *active* (minds-on) and *engaged* (not distracting), *meaningful* (applied to prior knowledge and transferred to the outside world), and occurring in a *socially interactive* environment.

Two additional characteristics of learning in playful contexts may also help explain why this pedagogical approach increases educational value: the joy and iteration that are inherent in play. Joy, or positive affect, has been linked to increased executive functions and academic outcomes (see Diamond, 2014 for a review) and even brain flexibility (Betzel et al., 2017). Iteration, or the mindful construction of new knowledge based on hypothesis testing and revising one’s own knowledge over time, is a hallmark of learning and play (Piaget, 1962). Each of these characteristics is supported by the learning literature and is inherent in playful learning contexts.

It is important to note that these characteristics align with learning across the play spectrum – from supporting the development of executive functions through free play (Elias and Berk, 2002) to the development of mathematics when playing games and engaging in guided play and/or exploration (see Ginsburg, 2009 for a review; e.g., Siegler and Ramani, 2008; DeCaro and Rittle-Johnson, 2012; Zosh et al., 2016). However, different types of play will embody the characteristics to different extents, which will then lead to different benefits for learning and other outcomes. For example, free play with friends may be high on joy and social interaction, which could lead to the development of socio-emotional skills. In contrast, guided discovery learning at a science museum may be high on iteration and meaning-making, which could support STEM learning. We argue that guided play particularly harnesses active, minds-on thinking, engagement, meaning-making, joy, and iteration more so than other types of play, which helps it maximize learning, particularly for academic skills.

### Active “Minds-On”

The study of early cognitive development centers on the idea that children play active roles in the construction of knowledge (e.g., Piaget, 1962). The activity, here though, that is crucial is that of *mental* activity – the active manipulation and processing of information rather than observation or rote responding. Active learning – where people are focused and engaged and where they are making decisions about the flow of incoming information – always outpaces passive learning where the information presented is merely meant to be absorbed. There is a rich and growing literature in this area.

While teaching new information directly may seem as if it has the advantage of being efficient, it may discourage further discovery, deeper processing, and ultimately, learning – leaving some researchers to dub this phenomenon the “double-edged sword” of pedagogy. Bonawitz et al. (2011) offer an excellent example of the power of active mental manipulation for learning. In their study, children were given the opportunity to play with and learn from a novel toy that had a number of non-obvious functions. In one condition, a knowledgeable adult demonstrated a subset of those functions and then children were allowed to play with the toy. In this case, children passively watched the knowledgeable adult and then were given the opportunity to play with and learn from the toy. In another condition, a non-knowledgeable adult “accidentally” demonstrated a hidden function, inspiring an active mindset for the children, and children were then again allowed to explore as they saw fit. Children in the first condition were less likely than children in the second condition to explore the toy and discover its additional features. Inspiring minds-on thinking led to discovery and learning. Yang and Shafto (2017) find computational evidence that this type of discovery-based, active learning is especially important when the teacher and learner have different assumptions and knowledge.

In other direct comparisons, Zosh et al. (2013) compared toddlers’ word learning when they were directly told the meaning of a novel word versus one in which they used process of elimination to determine the referent of a novel word. Even though the toddlers looked longer at the referent of the novel word in the first condition, they demonstrated greater retention of the novel label when they had to engage in the active processing task. Fisher et al. (2013) contrasted children’s ability to learn the identifying information for shapes (e.g., a triangle is any shape that has three connected sides regardless of whether they are symmetrical or not. It is not merely a shape with a point at the top). Four and five-year olds were shown examples of various triangles and asked to discover the secret of how they were related. Much like the word-learning example of Zosh et al. (2013), children who had to discover the information for themselves had better immediate and long-term (1 week later) retention of this information than children who were directly told.

As noted in the introduction, some researchers (e.g., Pellegrini) separate exploration from play. Here, we conceptualize exploration as minds-on thinking, either in playful or non-playful contexts. Exploration on its own does not make a context playful, but playful exploration represents minds-on-thinking in an enjoyable and child-directed context, and as such can help support learning. This is one reason that play in general, and guided play in particular, is so effective.

Active, minds-on thinking is intrinsic to play. When coupled with guidance toward a learning goal, in a playful setting, such as in guided play, it is more likely for children to be minds-on with the information that adults hope that they learn and this is more likely to be retained than information shared in more passive contexts.

### Engagement

Although being “minds on” is an important first step, staying “minds on” is crucial for learning. This is, perhaps, one of the greatest challenges that children face: Their ability to resist distraction and stay on task develops over childhood. Ruff and Lawson (1990) examined children’s sustained, focused attention during free play in childhood and found that children’s ability to maintain focused attention increased over the first 5 years. Kannass and Colombo (2007) found similar results in a comparison of children’s susceptibility to distraction between 3 to 4 years old. Further, children vary greatly in their susceptibility to distraction (Choudhury and Gorman, 2000; Dixon et al., 2006) and attention in earlier childhood is related to attention problems later in childhood (Martin et al., 2012). Even simple things such as pop-up books (Tare et al., 2010), instrumental music (Barr et al., 2010), and decorated classrooms (Fisher et al., 2014) distract young children and interfere with their learning. But crucially, susceptibility to distraction is, to some degree, malleable (Kannass et al., 2010; Neville et al., 2013).

Though play is often characterized as being a context with an absence of constraints, play naturally requires children to stay on-task, to balance their own wants with those of their social partners, and in the cases of pretend, to inhibit distractions from the immediate environment that conflict with the play narrative. As such, make-believe play has been linked to increased self-regulation ability but more data is necessary (see Berk and Meyers, 2013 for a review). For example, preschoolers who exhibited more socio-dramatic play early in the year showed increased self-regulation abilities later in the academic year (Elias and Berk, 2002). In a recent intervention study, Thibodeau et al. (2016) investigated the impact of a 5-week play-based intervention with preschoolers and found that those children who were in a fantastical pretend-play condition showed increased gains in executive function relative to children in a non-imaginative play condition or a business-as-usual control. This again speaks to the importance of a nuanced conceptualization of play. Not all play is created equal. Guided play in particular, where an adult scaffolds a situation toward a specific learning goal, may be especially helpful at maximizing engagement, particularly for younger children who are more susceptible to distraction.

### Meaningful

Meaningful information is that which is relevant, connected to something familiar, and able to be transferred to new situations or problems. For example, there is a difference between memorizing the fact that a triangle has three sides versus understanding that the pizza slices, tortilla chips, and sailboat sails in the real world resemble triangles.

The challenge of meaning-making is the work of the early years. Even a young child who, on the surface, knows the count list does not necessarily understand the principle of cardinality – this true knowledge unfolds over time (Wynn, 1990; Sarnecka and Carey, 2008). That is, knowing the word “three” is not synonymous with an understanding that the word “three” maps onto (or indicates) the quantity of three objects, and that sets of three things can come in diverse sets of things as varied as cups or books. A child might know that she is supposed to share toys with her brother because her mother has told her to, but not understand the reasons why (that her brother also wants to play with the toys and will be upset if he cannot). Similarly, being able to recognize the printed alphabet letters does not directly relate to the phonological awareness that is necessary for reading (Blair and Savage, 2006).

The distinction between surface and deeper learning has a long history in the scientific literature. From Einstein’s statement “*The value of an education … is not the learning of many facts but the training of the mind to think something that cannot be learned from textbooks*” to Ausubel’s (1968) distinction between rote versus meaningful learning, the idea that learning goes beyond basic content or knowledge to transferable, generalizable, deeper thought continues today. Shuell (1990) adds to this idea by stating that rote learning (e.g., knowing the count list or being able to recite the alphabet) is a precursor to “real” learning (e.g., having true numerical knowledge or being able to read) and this is expanded even more by Chi (2009) who emphasizes the use of previous knowledge to help actively construct new knowledge for conceptual change. Deeper learning in number or vocabulary requires that the learner not only store information, but also connect it to prior information (see Hadley and Dickinson, 2018, for an example in vocabulary development).

Comparing multiple examples and drawing analogies between situations and systems are some of the most powerful learning mechanisms available to young children. For example, children tend to rely on superficial surface properties when comparing objects unless they are given multiple examples. Seeing multiple examples prompts children to compare and examine the features that are common to each (Gentner and Namy, 1999). Making analogies between situations can also lead to new insights about problem-solving (e.g., Holyoak et al., 1984; Brown et al., 1986, 1989; Daehler and Chen, 1993; Chen, 1996) understanding scientific principles (e.g., Ganea et al., 2011; Kelemen et al., 2014; Shtulman et al., 2016), or learning moral lessons (see Mares and Woodard, 2005 for a review).

When children play, they choose themes, objects, and people that are relevant and interesting to them. Thus, they are motivated to make meaning out of the information in their play. Guided play or games can teach effectively by presenting information that is contextualized in ways that make sense to children. In one study, Habgood and Ainsworth (2011) created two versions of an educational computer game. In one version, 7- to 11-year-old children had to use an understanding of division to “divide” zombies and defeat them. In another version, children defeated the zombies using standard game methods, and then solved division problems at the end of each level. When the information about division and factors was made meaningful within the game, it led to better learning: Children who played the integrated version of the game outperformed the other group on a division test 2 weeks later.

Guided play may particularly support this type of meaning making because young children may struggle to do it on their own. Mares and Acosta (2008) found that kindergarteners who watched a story about dogs who befriended another dog with a missing leg tended to draw the very narrow lesson to “be kind to three-legged dogs,” rather than the broader moral lesson about accepting people who are different. However, children learn more from reading a book when a parent or other adult asks questions that encourage connecting the story to their existing knowledge – a process known as *dialogic reading* (e.g., Hargrave and Sénéchal, 2000). For example, the reader might ask children to think about how a character might be feeling or point out how an element in the story is similar to something from the child’s own life. Thus, adults can help scaffold children to make connections between new information and what they already know, thereby helping to make the new information more meaningful and supporting learning. This type of meaning-making supports learning in more informal, play-based contexts as well. For example, research in children’s museums suggests that instructing caregivers to ask questions such as “why?” helps children to learn more from their experience (Benjamin et al., 2010) and studies investigating how to increase learning pinpoint that scaffolding is crucial (Wolf and Wood, 2012; see Andre et al., 2017 for a review), especially to taking the learning beyond the museum. Guided play harnesses the power of children’s own agency and discovery but couples it with the adult-supported scaffolding that maximizes learning through meaning-making.

### Socially Interactive

Although children can play on their own, they also frequently play with parents, siblings, friends, or classmates. Playing with others also adds social meaning to the activity at hand. Chi (2009) describes how peer interactions can involve “building on each other’s contribution, defending and arguing a position, challenging and criticizing each other on the same concept or point, asking and answering each other’s questions” (p. 83). Through these processes, the two individuals each contribute to the conversation in such a way that it helps construct new shared knowledge. Indeed, it has been suggested that the sharing of information between individuals acts as a type of “natural pedagogy” (Csibra and Gergely, 2009, p. 148), in other words, social interaction is, in itself, a mechanism for learning.

Entire theories are centered around the role and importance of social partners not just for learning but for lifetime attainment of things such as independence, self-worth, and fulfillment (e.g., Vygotsky, 1967). Perhaps nowhere is this more important than in infancy and early childhood, and infants seem to be born looking for this interaction (e.g., Meltzoff and Moore, 1983). Infants and children prioritize input and learn more from social cues compared to non-social presentations of the same information [e.g., a human arm versus a robotic arm (Wu et al., 2011); a face or a flashing cue (Wu and Kirkham, 2010), and even a communicative point versus non-communicative reaching (Yoon et al., 2008)].

Social interaction in infancy and childhood centers around interactions with parents/caregivers and peers^1^. Both have been shown to be important resources for children. Parents and/or caregivers are an infant’s initial social partner, and the quality of this early caregiver-infant relationship has been linked to many different positive outcomes. For example, a parent’s contingent responses to a child’s vocal play support language development (see Tamis-LeMonda et al., 2014 and Reed et al., 2016 for reviews). Recent work suggests that direct gaze sharing between a parent and infant promotes neural connectivity and communication bidirectionally (Leong et al., 2017).

Parent/child interaction can also promote healthy socioemotional regulation critical for academic achievement and can even serve as a protective factor against the negative physical and cognitive effects of stress (see Center on the Developing Child at Harvard University, 2016 for a review; Nelson et al., 2014; Nelson, 2017).

Play encourages social interaction for young children in a number of ways. Playing with peers has been shown to support learning. For example, Ramani (2012) found that children built larger, more complicated structures when they were engaged with a peer in a playful building activity compared to when they were presented with the same materials in an adult-directed and adult-structured activity. Similarly, social interaction among preschoolers was related to increased complexity of building with blocks (Trawick-Smith et al., 2017). Although Park and Lee (2015) suggest that one of the advantages of working with a peer is benefiting from a higher-ability peer or one with higher social skills, even the illusion of working collaboratively has positive effects. Preschoolers who were told they were collaboratively working on a puzzle with a child in the next room persisted longer on the task and reported liking it more compared to children who knew they were working alone or were told that they were taking turns (Butler and Walton, 2013). And crucially, children seem to be rather discerning and take into account the knowledge and reliability of their social partners (Bonawitz and Shafto, 2016).

While free play has traditionally been recognized as optimal for promoting social interaction, even in play with peers, it is important for adults to scaffold and protect the playful peer interaction (Ghafouri and Wien, 2005) as even young children are susceptible to social loafing (Arterberry et al., 2007), bullying (Kirves and Sajaniemi, 2012), and exclusion (Fanger et al., 2012), suggesting that guided play may have a role in the development of positive social skills.

It is important to note that the presence of social interaction does not necessarily make a situation playful. Teachers using didactic methods to instruct a class can be interacting with a class that is devoid of any play. Further, and on the opposite side, children can engage in solo play that is joyful and child directed, but that is not social at all. We suggest here that playful pedagogies are effective because they often harness the power of high quality social interaction, *in combination with* the other characteristics outlined here (joy, active thinking, engagement, meaningful, and iterative) to support learning^2^.

### Iterative

Acquiring knowledge requires more than the deposit of facts from the more educated into the less educated; instead, learning is similar to the scientific process. As Piaget (1964) notes:

Knowledge is not a copy of reality. To know an object, to know an event, is not simply to look at it and make a mental copy or image of it. To know an object is to act on it. To know is to modify, to transform the object, and to understand the process of this transformation, and as a consequence to understand the way the object is constructed. (p. 176)

To learn, even young infants, or, as Gopnik et al. (1999) called them, the “scientists in the crib,” engage in the process of generating hypotheses, testing those hypotheses, and then using the generated data to inform one’s own understanding. In other words, they construct the knowledge using the methods described by Piaget. Learning requires that knowledge generation is an *iterative* process in which a child uses what he or she knows to generate new hypotheses, tests those hypotheses using minds-on thinking, and updates his or her understanding based on those tests. A striking example of this comes from decades of research examining young infants’ reasoning about physical objects and relationships finding that even young infants have expectations about what objects can and cannot do, but they revise this knowledge over infancy and it becomes more accurate and nuanced as they acquire additional experience (see Baillargeon, 2004 for a review; Wang et al., 2016; Baillargeon and DeJong, 2017).

Indeed, children explore more when violations of their expectations occur (e.g., Schulz and Bonawitz, 2007; van Schijndel et al., 2015). In Stahl and Feigenson (2015), researchers presented 11-month-old infants with visual presentations in which expectations about normal objects were violated (e.g., an object passed through a solid surface or an object seemingly blipped out of existence) and compared their immediate learning to presentations in which there were no violations of expectations. The infants who observed an object appear to violate physical laws were more likely to learn about a hidden property of the object, and they spent more time exploring the objects. They even appeared to test out the apparent violation; for example, children who observed an object appear to pass through a solid wall spent more time banging it on surfaces than children who did not witness the violation. Preschoolers will preferentially explore a toy characterized by confounded evidence over toys without ambiguity (Schulz and Bonawitz, 2007). Thus, not only do young infants generate rules based on evidence but they actively seek to revise these rules over time.

Play inspires iteration. Guided play, in particular, can be described as “constrained tinkering” where, within a bounded exploration space, children have the freedom to test out different hypotheses. Unlike more direct instruction contexts in which active exploration and discovery are often thwarted, playful contexts encourage exploration and discovery as a focus. For example, in one study, children were more likely to play with a toy when the causal structure of the toy (i.e., which lever caused a toy to pop up) was ambiguous than when it was clearly demonstrated to them (Schulz and Bonawitz, 2007; see also Cook et al., 2011; Buchsbaum et al., 2012). Pretend play also invites iterative processing as children must not only keep in mind conceptual premises that exist outside of reality but also adapt to changing circumstances as the play session continues (e.g., Harris and Kavanaugh, 1993; Weisberg and Gopnik, 2013). As with the other characteristics, iteration alone is not a necessary feature for play. Yet, play often inspires iteration. And although all types of play may inspire simple iteration, some adult support in the form of guided play may be necessary for more advanced types of hypothesis testing, such as those involved in higher scientific thinking (e.g., generating hypothesis about what variables cause a particular effect and testing those hypotheses in the midst of confounding variables). Research has found that children are not very good at designing appropriate experiments on their own (e.g., Klahr et al., 1993), but can do so in a child-directed and fun way if offered some adult guidance (see Lazonder and Harmsen, 2016 for a meta-analysis).

### Joyful

Joy is an essential element of play: Early scientific writings on play mention “positive affect” and “intrinsic motivation” as defining features of what makes an activity playful (Krasnor and Pepler, 1980). Joy is inherent, and required, for an activity to be considered play. Even in the most constrained definitions of play cited above, joy is a central characteristic.

The idea that positive affect influences cognition is not new (Isen, 1984). Ashby et al. (1999) proposed a neuropsychological theory relating positive affect to both long-term and working memory as well as creativity in problem solving. Indeed, positive affect is linked to increased creativity (Isen et al., 1987), and creative thinking is linked to increased learning (Resnick, 2007; Zosh et al., 2017).

The idea that emotions and cognition are linked is only growing in popularity. Fischer and Bidell (2006) highlight the dynamic nature of development, with emotion and cognition as “two sides of the same coin as characteristics of control systems for human activity. Emotion is together with cognition at the center of mind and activity.” (p. 370). Recent research in psychology and neuroscience furthers supports this idea (Immordino-Yang and Damasio, 2007). In fact, an entire field of psychology touts its benefits for a variety of positive outcomes, including learning (Seligman, 2002).

Positive affect is not the only aspect of joy implicated in learning. Surprise also seems to play a role in increasing curiosity and exploration – leading to increased learning potential. In the Stahl and Feigenson (2015) study described above, infants learned more when their expectations were violated, and also engaged in more information-seeking behavior and hypothesis-testing, congruent with the violations they observed. Neuroscientists are beginning to unravel the neural correlates of affect and surprise on learning (Betzel et al., 2017), potentially through increased dopamine levels, which are implicated in the brain’s reward system and motivation (e.g., Cools, 2011; Dang et al., 2012).

Beyond positive affect, intrinsic motivation is a key distinguishing feature of play, even in the traditional definitions offered above. The definition of intrinsic motivation offered by Ryan and Deci (2000) overlaps considerably with our conceptualization of play.

Perhaps no single phenomenon reflects the positive potential of human nature as much as intrinsic motivation, the inherent tendency to seek out novelty and challenges, to extend and exercise one’s capacities, to explore, and to learn…. The construct of intrinsic motivation describes this natural inclination toward assimilation, mastery, spontaneous interest, and exploration that is so essential to cognitive and social development and that represents a principal source of enjoyment and vitality throughout life (Csikszentmihalyi and Rathunde, 1993; Ryan, 1995) (Ryan and Deci, 2000, p. 70).

This definition stresses minds-on thinking, engagement in the material to be learned, exploration/iterative thinking, assimilation (meaningfulness), and learning. These concepts all align with the same exact features that support learning. The key here, however, is that children engage in this process with agency. They are intrinsically motivated to learn and discover. Playful learning contexts, in which children lead the play experience with or without adult support (see **Figure 1**), thus capitalize on this intrinsic motivation to harness children’s own learning potential. Decades of research have investigated the role of intrinsic motivation and support its importance for learning and creativity among other positive outcomes (Ryan and Deci, 2017). In a recent review of programs that improved children’s executive functions, Diamond (2012) highlighted a potential mechanistic explanation for why play and learning may be mutually supportive: “Children devote time and effort to activities they love; therefore, EF interventions might use children’s motivation to advantage” (p. 335). Play, an inherently positive experience for children, has the potential to be the context that provides this advantage.

### Outstanding Issues

Active, engaged, meaningful, social, iterative and joyful are characteristics that individually and collectively appear in a number of scientific articles that highlight processes involved in optimal learning. These same characteristics coalesce in play. Thus, playful learning – and in particular guided play – should confer real learning advantages for academic and social outcomes.

Adopting a more nuanced understanding of the play construct allows us to better understand how play might support learning: Different types of play may be optimal for different types of learning. This speaks not only to the theory of why guided play works, but also to long-standing debates in the field regarding optimal pedagogical approaches to learning. It also raises new questions that can guide further research.

To the issue of why guided play works, we not only offer the parallel between the characteristics of play and high-quality learning, but also a theoretical argument for why guided play, in particular, feeds learning specific information. Bonawitz et al. (2009) argue that the possibility space of learning new information is vast, “Learning the affordances of a novel artifact is challenging because for any object, there are an unknown, and potentially large, number of causal properties.” (p. 1575). However, the danger of direct pedagogy is that it limits exploration and discovery, “…in natural learning contexts, pedagogical demonstrations cannot demonstrate all there is to know, and teaching will necessarily be limited.” (p. 1580). Because there are too many degrees of freedom in a free play situation, a child actively engaged with shapes, for example, who is not “guided” toward a learning outcome could guess that triangles have “points on top,” are in “primary colors,” or are “2 inches in length” rather than focusing on key variables like the number of sides and angles. However, what direct instruction does is teach children that these exact exemplars are triangles and the child may not understand that a square split along its diagonal is triangle because that was not what was taught. Thus, when free play pedagogies have been compared to direct instruction pedagogies – direct instruction pedagogical approaches are often better suited to learning (Pianta et al., 2009; Fuller et al., 2017). Bonawitz et al. (2009) suggest “Understanding how to combine the efficiency of pedagogical knowledge transmission while encouraging curiosity and exploratory play is an important direction for future work.” (p. 1580).

The introduction of a play spectrum with nuanced categories like guided play, however, changes the dynamic and answers this call. Guided play, like direct instruction techniques, constrains the contexts in which children generate hypotheses, effectively helping them to hone in on the learning and avoid distraction. For example, it invites children to play with a set of triangles that can be compared and contrasted such that key properties “fall out” of the context. It might also offer a “coach” who helps children direct attention to these defining characteristics. Thus, in Bonawitz’s theory, guided play points children in a direction that allows for “constrained tinkering.”

Guided play, however, also adopts the characteristics noted above and allows or even motivates the child to direct the learning in a joyful way. Thus, guided play, sitting midway between direct instruction and free play, allows for the best of both pedagogical approaches. In this context, it no longer makes sense to say that pedagogies should be either play or direct instruction. High quality schools can have rich curricular goals and at the same time deliver them through guided play techniques. Indeed, this is precisely the formula that was recommended in a number of recent papers (Bustamante et al., 2017; Fuller et al., 2017; Jenkins and Duncan, 2017), and Jenkins and Duncan (2017) write about the most effective pre-K curricula, “… these curricula provide teachers with lesson plans to follow in which playful activities are strategically organized to present children with learning opportunities that are focused, sequential and cumulative” (p. 39, see also Burchinal, 2018).

By recognizing a continuum of play categories, we can better understand why play in general, and guided play in particular, is related to learning and we can accelerate learning outcomes by designing targeted play pedagogies.

This spectrum-based view of play also allows us to better formulate questions about where and when particular types of playful learning might prove predictive of particular outcomes. As Jirout and Klahr (2012) argue, for second grade math curricula, direct instruction might prove a more effective way to help children settle on the right formulas (though see Weisberg et al., 2016). Might dramatic play be an optimal way for young children to learn socioemotional skills (Copple and Bredekamp, 2009; Goldstein and Lerner, 2017; but see Lillard et al., 2013)? Might guided play lead to stronger outcomes in literacy (Han et al., 2010; Hassinger-Das et al., 2016; Cavanaugh et al., 2017; Toub et al., 2018) and STEM [e.g., spatial thinking (Fisher et al., 2013)]? While there are hints in the literature that confirm each of these hypotheses, more work needs to be done. Indeed, this work is beginning. In an impressive review and analysis of pretend play in particular, Lillard et al. (2013) explore whether or not pretend play holds a causal role in supporting development. They find that when carefully examined, the evidence to date does not allow us to draw any firm conclusions about the casual role of pretend play and suggest that more and better research is needed. We could not agree more and suggest that viewing play as a spectrum allows us to create new hypotheses and design new studies to help tease apart the role of play and playful learning in developing a whole host of skills across childhood and beyond. In fact, Lillard et al. (2013) even directly state that the lack of firm research about the impact of pretend play on development does not equate to a call for teacher-centered approaches to education and learning. Instead, “The hands-on, child-driven educational methods sometimes referred to as “playful learning” (Hirsh-Pasek et al., 2009) are the most positive means yet known to help young children’s development.” (Lillard et al., 2013, pp. 27–28).

That is, it is possible that as we sketch out a suite of 21st century skills like those suggested by Golinkoff and Hirsh-Pasek (2016) that different types of playful learning are more or less effective. It will also be critical to explore whether different types of play afford these different advantages in the same way across context and time. As Schindler et al. (2017) reminds us,

“This rapidly advancing science calls for a new early childhood agenda that builds on current investments in quality improvement and system building and seeks new models and methods in the quest for greater impacts. To this end, there is a need for enhanced theories of change and more effective strategies that move beyond the general question of “what works?” and seek a more nuanced understanding of what works (and what does not) for whom and why, and in what contexts (Shonkoff and Fisher, 2013)” (p. 1436).

## Conclusion

While many would agree that play is an important part of childhood and supports social interaction and growth, questions about the relationship between play and learning abound and there is renewed energy around the study of play. To better harness this energy, though, we need to have a working definition of play that is not as broadly construed as that proposed in the global literature. Here, based on the newest research and with respect to playful learning studies in the past, we propose a multidimensional definition of play that creates a spectrum of play opportunities from free play through guided play to games and then playful direct instruction (a form of direct instruction with minor playful elements to try to keep children engaged). This more nuanced definition allows us to better define the mechanisms for playful learning – how and why different types of play are related to various types of outcomes. It also challenges us to raise new questions in the field that should enhance our understanding of how play relates to varied outcomes across time and in varied contexts.

## Author Contributions

JZ was responsible for the first draft of the manuscript. KH-P and JZ were primarily responsible for main revisions. EH, HJ, CL, DN, SS, and DW were responsible for writing sections of the manuscript. All authors contributed to manuscript revision, read and approved the submitted version.

## Conflict of Interest Statement

The authors declare that the research was conducted in the absence of any commercial or financial relationships that could be construed as a potential conflict of interest.

## Footnotes

1 Note that parasocial relationships, in which children form emotionally connected relationships with characters, also have been linked to increased learning potential. See Calvert (2017) and Hirsh-Pasek et al. (2015) for reviews of how parasocial relationships can utilize the benefits of social interaction to maximize learning.

2 Note that not all of the examples provided in this section would necessarily fall somewhere along our playful continuum (e.g., watching a video). Instead, what we suggest is that social interaction, in general, has the power to support learning and that, when combined with the other characteristics, helps explain why playful pedagogies are so effective.
